# Circular RNA Circ-0002570 Accelerates Cancer Progression by Regulating VCAN *via* MiR-587 in Gastric Cancer

This article has been retracted.

**DOI:** 10.3389/fonc.2021.733745

**Published:** 2021-10-06

**Authors:** Lei Yang, Yong-ning Zhou, Miao-miao Zeng, Nan Zhou, Bin-sheng Wang, Bo Li, Xiao-liang Zhu, Quan-lin Guan, Chen Chai

**Affiliations:** ^1^ Department of General Surgery, The First Hospital of Lanzhou University, Lanzhou, China; ^2^ Department of Gastroenterology, The First hospital of Lanzhou University, Lanzhou, China; ^3^ Department of Oncology, The First Hospital of Lanzhou University, Lanzhou, China; ^4^ Department of Surgical Oncology, The First hospital of Lanzhou University, Lanzhou, China; ^5^ Department of General Surgery, The People’s Hospital of Suzhou New District (SND), Suzhou, China

**Keywords:** circ-0002570, circular RNA, miR-587, VCAN, metastasis, biomarker

## Abstract

**Background:**

Circular RNAs (circRNAs) are closely associated with the occurrences and progress of gastric cancer (GC). We aimed to delve into the function and pathological mechanism of Circular RNA-0002570 (circ-0002570) in GC progression.

**Methods:**

CircRNAs differentially expressed in GC were screened using bioinformatics technology. The expression of circ-0002570 was detected in GC specimens and cells *via* qRT-PCR, and the prognostic values of circ-0002570 were determined. The functional roles of circ-0002570 on proliferation, migration, and invasion in GC cells were explored *in vitro* and *in vivo*. Interaction of circ-0002570, miR-587, and VCAN was confirmed by dual-luciferase reporter assays, Western blotting, and rescue experiments.

**Results:**

Circ-0002570 expression was distinctly increased in GC tissues compared to adjacent normal specimens, and GC patients with higher circ-0002570 expressions displayed a short survival. Functionally, knockdown of circ-0002570 resulted in the inhibition of cell proliferation, migration, and invasion, and suppressed tumor growth *in vivo*. Mechanistically, miR-587 was sponged by circ-0002570. VCAN expression in NSCLC was directly inhibited by miR-587. Overexpression of circ-0002570 prevented VCAN from miR-587-mediated degradation and thus facilitated GC progression.

**Conclusion:**

The circ-0002570-miR-587-VCAN regulatory pathway promoted the progression of GC. Our findings provided potential new targets for the diagnosis and therapy of GC.

## Introduction

Worldwide, gastric cancer (GC), the second leading cause of tumor-associated mortality, is the fourth most common cancer and is associated with high morbidity (1). The incidence and mortality of GC in China have been increasing in the last 20 years (2). Although great progresses have been made in the early screening and treatments of GC with the clinical application of adjuvant chemotherapy and/or surgical operation, the clinical outcome of many patients remains unfavorable. GC patients with advanced stages are incurable and have a poor 5-year overall survival rate of nearly 5% (3, 4). Thus, for early screening and novel treatments of GC patients, figuring out its molecular mechanisms and exploring novel and sensitive biomarkers are critical.

Circular RNAs (circRNAs) are known as a certain class of non-coding RNAs, forming a covalently closed continuous loop *via* back-splice without 3’-end or 5’-end (5). Previously, it was considered that aberrant splicing processes generate them (junk) without any biological functions (6). In recent years, with the development of high-throughput sequencing, more and more circRNAs are demonstrated to be abnormally expressed in different cells and specimens, indicating that they could exhibit specific biological functions (7, 8). In addition, more and more evidences have confirmed that circRNAs exhibited regulatory effects on the tumorigenesis and metastasis of different types of tumors and would be novel diagnostic biomarkers and therapeutic targets (9, 10). Besides, circRNAs have been functionally identified to act as a miRNA sponge and then modulate the expression of human genes, which results in their participation in the tumor progression (11, 12). However, to date, only a small portion of lncRNAs are functionally identified.

Circular RNA-0002570 (circ-0002570) was a newly identified circRNA. Recently, Liu and his group firstly identified circ-0002570 as a diabetic retinopathy-related circRNA that can sponge miR-1243 (13). However, whether circ-0002570 was dysregulated in tumors, and its potential function have not been investigated. In this research, our group firstly provided evidence that circ-0002570 was highly expressed in GC. Then, we further explored the possible function of circ-0002570 in GC progression. Our findings revealed that circ-0002570 was a novel biomarker and therapeutic target for GC patients

## Patients and Methods

### Sample Collection

A total of 24 GC tissues and paired adjacent noncancerous tissues were collected from The First Hospital of Lanzhou University between January 2018 and July 2019, and this study was approved by the First Hospital of Lanzhou University Ethics Committee. Tissues of patients confirmed to be GC by pathology were immediately chilled in tissue nitrogen. Preoperative treatment for cancers was not used for all patients. All participants were informed and signed the informed consent form for this study.

### Cell Culture

Human normal gastric mucosal cells (GSE-1) and GC cell lines (AGS, MKN28, MKN45, SGC7901, HGC27, and BGC23) were obtained from the Central Culture Collection of the Chinese Academy of Sciences (Shanghai, China). The cells were cultured in DMEM medium (Jinuo Biology, Hangzhou, Zhejiang, China). In a 37°C, 5% CO_2_ incubator, subculture was carried out.

### Transfection

Circ-0002570 shRNA (circ-0002570-sh-#1 and circ-0002570-sh-#2), VCAN pcDNA, miR-587 inhibitor, miR-587 mimics, shRNA NC (sh-NC), inhibitor NC, mimic NC, and NC vectors were purchased from Sangon Bioengineering (Shanghai, Pudong, China). AGS and SGC7901 cells were transfected with siRNAs, miRNA, or the plasmid vectors based on the Manufacturer Directory. RT-qPCR and Western blot assays were applied to confirm transfection efficiency

### Bioinformatics Analysis

Firebrowse (http://firebrowse.org/) was used to download The Cancer Genome Atlas (TCGA) stomach adenocarcinoma(STAD) sequencing and clinical data. In the NCBI web server, we downloaded microarray data (GEO: GSE83521). The web tool Kaplan–Meier Plotter (http://kmplot.com/analysis/index.php?p=service&cancer=gastric) was used for survival assays of GC patients. Outdo Biotech (Shanghai, China) (Outdo cohort) provided a tissue microarray (TMA) cohort containing a total of 104 GC and adjacent non-tumor specimens. R (version 3.4.3) (https://www.r-project.org/) was applied for subsequent assays. Differentially expressed circRNAs were chosen based on the following criteria: fold change > 2 and *p* < 0.05. On the top 30 differentially expressed circRNAs, the hierarchical clustering analysis was conducted. circBank (http://www.circbank.cn/) and CircInteractome (https://circinteractome.nia.nih.gov/) were applied to predict the miRNA-binding sites of circ-0002570. TargetScan (http://www.targetscan.org/vert_72/) and Starbase (http://starbase.sysu.edu.cn/) were used to predict the target of miR-587. GSEA v3.0 software was applied to analyze mRNA expression data. Package “GSVA” in R was used to perform GSVA analysis for assays of the change of pathway enrichment. GO genome and KEGG pathway genome were applied for the conduction of the genome enrichment analysis.

### RNA Isolation and Quantitative Real-Time PCR

TRIzol reagent (Aobolai Biology, Haidian, Beijing, China) was used for the extraction of RNA in cells and specimen samples based on manufacturer directory. cDNA was synthesized using the PrimeScript RT Reagent Kit (Takara, Hangzhou, Zhejiang, China). SYBR Green Realtime PCR Master Mix was applied to conduct RT-PCR assays on the Applied Biosystems 7300 Real Time PCR system. The relative expression of all factors were examined using 2^−ΔΔCt^ methods. GAPDH and U6 were normalized as endogenous controls. The primers are shown in **Table 1**.

**Table 1:** The primers used in this study for RT-PCR.

Names	Sequences (5’-3’)
hsa_circ_0002570: Forward	CAAGCTCTGACCTTTCGCAA
hsa_circ_0002570: Reverse	AGCCACCGGAGAAAATTTGA
VCAN: Forward	GTAACCCATGCGCTACATAAAGT
VCAN: Reverse	GGCAAAGTAGGCATCGTTGAAA
miR-587: Forward	CTCAACTGGTGTCGTGGAGTCG
	GCAATTCAGTTGAGGTGACTCA
miR-587: Reverse	ACACTCCAGCTGGGTTTCCATAGGTGATG
GAPDH: Forward	GGAGCGAGATCCCTCCAAAAT
GAPDH: Reverse	GGCTGTTGTCATACTTCTCATGG
U6: Forward	GCGCGTCGTGAAGCGTTC
U6: Reverse	GTGCAGGGTCCGAGGT

### RNase R Digestion

At 37°C with 3 U/μg of RNase R (Biovision, Amyjet, Wuhan, China), total RNAs (8 μg) were incubated for 20 min. According to previously published procedures, the RNase R digestion reaction was conducted twice (14).

### Cell Counting Kit-8 Assays

The AGS and SGC7901 cells were seeded in 96-well plates for examining proliferation ability by CCK-8 assays (Dojindo, Nanjing, Jiangsu, China). Then, 15 μl of CCK8 solution was added. A Thermo-max microplate reader was applied to examine the absorbance at 450 nm.

### Colony Formation Assay

In brief, transfected AGS and SGC7901 cells were seeded onto six-well plates (1,000 cells/well). After the cellular culture for 14 days, 0.1% crystal violet was applied to stain the plates. Subsequently, PBS (YiTabio, Pinggu, Beijing, China) was used to wash the plates three times. Colonies with at least 50 cells were counted manually.

### 5-Ethynyl-2’-Deoxyuridine Staining

Twenty-four hours after circ-0002570 knockout in AGS and SGC7901 cells with shRNAs, Click-iT EdU staining kit (Bio-rad, Yihui Biology, Shanghai, China) was applied to stain the AGS and SGC7901 cells according to the specific procedures in the kit instructions. Finally, the number of EDU-positive cells was detected by fluorescence microscopy.

### TUNEL Assay

Cell apoptosis was examined through TUNEL staining assays. AGS and SGC7901 cells were fixed in 4% paraformaldehyde for 15 min. The *In Situ* Cell Death Detection Kit, POD (Roche, Shenzhen, Guangdong, China), was applied to stain the collected cells based on the manufacturer’s protocol. Relative fluorescence intensity was detected *via* an EVOS FL microscope (Invitrogen).

### Cell Scratch-Wound Assay

AGS and SGC7901 cells (1 × 10^6^) were seeded into each well supplemented with 2 ml of complete medium. At the center of the well plate, a vertical scratching mark was made until the cells spread across the bottom of the plate. The cells were washed with PBS twice to remove the cell debris. At different time points (0 and 48 h), observation of the cells in plates was carried out using a microscope. Image Pro-Plus 5.0 software was applied to examine the width of the wound.

### Transwell Assay

Transwell chambers (Corning, Haidian, Beijing, China) were used to perform cell culture for migration and invasion assays. Diluted Matrigel (BD Biosciences, Guangzhou, Guangdong, China) was applied to coat the insert membranes for invasion assays. Cells (5 × 10^4^) were added to the upper chamber and cultured for 48 h. After 24 h of incubation, the invaded cells were fixed with 4% paraformaldehyde and stained with Giemsa, while the cells on the upper surfaces were scraped. The number of cells on the lower surface was then counted under a light microscope.

### Tumor Xenograft *In Vivo*

AGS and SGC7901 cells (4 × 10^4^) were injected into female BALB/c-nu nude mice (weighing 15–20 g, Shanghai SIPPR-BK Laboratory Animal). Each group (circ-0002570-sh group and NC-sh group) had five mice. Tumor sizes were assessed once per week by a digital caliper. After 28 days, the mice were decapitated, followed by the collection of the tumors. Immunohistochemistry was performed on tumor tissues for Ki-67 as previously described (15). The tumor volumes were recorded every one week and calculated by the use of a formula (length × width^2^ × 0.5). The animal studies were approved by the Institutional Animal Care and Use Committee of The First Hospital of Lanzhou University, and were performed according to institutional guidelines.

### RNA Fluorescence *In Situ* Hybridization

FISH assays were performed as described previously (16).

### Luciferase Reporter Assay

The wild-type (WT) sequence of the circ-0002570 together with the WT 3’UTR sequence of the VCAN containing predicted binding site of the miR-587 were amplified. Then, the collected sequences were subcloned into the luciferase reporter vector pGL3-basic (Promega) (Promega, Shenzhen, Guangdong, China). Quick Change Lightning kit (Stratagene, Hangzhou, Zhejiang, China) was adopted for the construction of mutant-type (MUT) sequence of the circ-0002570 and VCAN. AGS and SGC7901 cells received the transfection procedure using the pGL3-circ-0002570-MUT, pGL3-circ-0002570-WT, or pGL3-VCAN 3’UTR, together with the miR-587 mimics or the matched controls. A Dual-Luciferase Assay Kit (Promega) was used to detect the luciferase activity.

### RNA Immunoprecipitation Assays

RIP assays were performed as described previously (17).

### Western Blot Assays

In RIPA buffer with 1% PMSF, cultured cells were lysed. Protein was loaded and separated by SDS-PAGE gel and transferred onto PVDF membrane. Primary antibodies were applied to probe the blots at 4°C, followed by incubation of HRP-conjugated secondary antibodies. ECL substrates (Pierce) were used for the visualization of signals. Using densitometry analysis in Quantity One software (Bio-Rad, USA), the protein bands were quantified. GAPDH was used as an endogenous control. Primary antibodies include VCAN (1:1,000, ab19345, Abcam, MA, USA) and GAPDH (1:1,000, ab9485, Abcam, MA, USA).

### Statistical Analysis

R language (version 3.5.2) and GraphPad Prism software (version 8.0.1) were applied for statistical analyses. Data from three independent experiments were shown as mean ± standard deviation (SD), followed by Student’s *t*-test or one-way analysis of variance (ANOVA). Kaplan–Meier curves were applied to perform survival analysis, followed by the log-rank test calculating *p*-values. All *p*-values < 0.05 were considered significant.

## Results

### The Identification of Dysregulated CircRNAs and Characterization of Circ-0002570 GC

To examine the dysregulated expressed circRNAs between tumor and normal gastric specimens, our group conducted hierarchical clustering analysis. The top 30 dysregulated circRNAs of GSE83521 were shown in the heat map, and circ-0002570 was one of the most upregulated circRNA in GC (**Figure 1A**). Circ-0002570 is derived from the FAM73A gene located on 1p31.1, resulting from back-splicing of exons 3, 4, 5, 6, and 7. The back-splicing junctions of circ-0002570 were demonstrated by the use of Sanger sequencing (**Figure 1B**). RT-PCR assays demonstrated divergent primers can amplify the circ-0002570 from cDNA, but not from gDNA (**Figure 1C**). Moreover, we found that compared with FAM73A, circ-0002570 was significantly resistant to RNase R, implying that circ-0002570 was a circRNA (**Figure 1D**). RT-PCR revealed that circ-0002570 expression was distinctly increased in GC specimens compared with the matched normal specimens (**Figure 1E**). Similarly, circ-0002570 expressions were also increased in six GC cell lines compared with GSE-1 (**Figure 1F**). According to ISH levels of circ-0002570 using Outdo TMA cohort, we found that high circ-0002570 expression in GC patients was a frequent event (**Figures 2A, B**). Clinical assays revealed that patients in high-circ-0002570 expressing group had a shorter overall survival than those in low-circ-0002570 expressing group (**Figure 2C**).

**Figure 1:** Circ-0002570 expression was distinctly increased in GC. **(A)** The Heatmap was drawn to show the differentially expressed circRNAs in GC tissues by analyzing the GSE31210. **(B)** Sanger sequencing was applied to demonstrate the back splicing junction. **(C)** RT-PCR and gel electrophoresis were performed to check the existence of circ-0002570. Circ-0002570 can only be amplified in cDNA. **(D)** The relative levels of FAM73A and circ-0002570 were examined by RT-PCR after treatments with RNase R or mock in AGS and SGC7901 cells. **(E)** RT-PCR for the expression of circ-0002570 in 24 pairs of GC specimens and non-tumor specimens. **(F)** The levels of circ-0002570 in six GC cells and GSE-1 cells were determined by RT-PCR. *p < 0.05, **p < 0.01, ***p < 0.001. ns, no significant.

**Figure 2:** The expressing pattern of circ-0002570 in GC specimens and normal gastric specimens, and its clinical significance. **(A, B)** Percentage of circ-0002570 ISH levels in normal specimens (*n* = 76) and GC specimens (*n* = 104). **(C)** Survival assays based on circ-0002570 expression in 104 patients from Outdo TMA cohort. ***p < 0.001.

### Knockdown of Circ-0002570 Suppressed the Proliferation and Metastasis of GC Cells

To delve into the functions of circ-0002570 on the functions of GC cells, a circ-0002570-knockdown expressing model was successfully constructed and demonstrated by the application of qRT-PCR (**Figure 3A**). The expression of FAM73A remains unchanged in AGS and SGC7901 cells (**Figure 3B**). CCK-8 assay showed that the OD450 values at 72 h post-culturing were distinctly reduced in the sh-circ-0002570 group compared with NC-sh group (**Figure 3C**). Edu and Colony formation assays also revealed that silence of circ-0002570 suppressed the proliferation of AGS and SGC7901 cells (**Figures 3D, E**). Scratch wound assays suggested that the invasive and migratory capacities of AGS and SGC7901 cells were also repressed in circ-0002570-sh transfected GC cells (**Figure 3F**). Transwell assays revealed that the number of migrative and invasive cells in the circ-0002570-sh-transfected sample also significantly decreased compared with the control transfectants (**Figures 3G, H**). TUNEL assays showed that circ-0002570 knockdown significantly promoted cell apoptosis (**Figure 3I**). According to the results of *in vivo* using Xenografts model, our group found that the tumor growth of nude mice with circ-0002570 knockdown speed was slower than the NC-sh group (**Figure 4A**). In addition, it was found that the tumor volume and weight were distinctly lessened in the circ-0002570-sh group compared with the NC-sh group (**Figures 4B, C**). In the collected tumor specimens, circ-0002570 expression was distinctly downregulated in the circ-0002570-sh group compared with the NC-sh group (**Figure 4D**). In addition, as displayed in **Figure 4E**, the positivity of Ki-67 was reduced by silenced circ-0002570. Taken together, these findings indicated that circ-0002570 enhanced carcinogenesis of GC cells.

**Figure 3:** The oncogenic roles of circ-0002570 in the progression of GC cells. **(A, B)** RT-PCR determined the expression of circ-0002570 and FAM73A in AGS and SGC7901 cells transfected with NC-sh, circ-0002570-sh#1, or circ-0002570-sh#2. **(C)** CCK-8 assay presented the proliferation of AGS and SGC7901 cells transfected with NC-sh or circ-0002570-sh. **(D)** Edu assays determined the proliferative ability. **(E)** Colony formation assay in AGS and SGC7901 cells after circ-0002570 knockdown. **(F)** Migration of AGS and SGC7901 cells in different transfection groups was detected by scratch wound assays. **(G, H)** The migrative and invasive capacity of NC-sh or circ-0002570-sh transfected AGS and SGC7901 cells was assessed by transwell assays. **(I)** TUNEL was employed to analyze the apoptotic index. *p < 0.05, **p < 0.01, ***p < 0.001.

**Figure 4:** Knockdown of circ-0002570 accelerates tumorigenesis *in vivo*. **(A)** Tumors derived from mice in two different groups were presented. **(B, C)** Tumor weight and volume were detected in tumor tissues of nude mice injected with circ-0002570-sh transfected AGS cells. **(D)** RT-PCR for the expression of circ-0002570 in the collect tumor samples. **(E)** HE staining and IHC staining of Ki-67 in two groups. ***p < 0.0001.

### Circ-0002570 Functions as a Sponge for MiR-587

Then, we examined the subcellular localization of circ-0002570 given that the function of one lncRNA depended on its subcellular distribution. Using FISH, we observed that circ-0002570 was expressed in both the nucleus and cytoplasm (**Figure 5A**). By searching online databases (circBank and CircInteractome), our group screened two miRNAs (miR-587 and miR-935), which are hypothesized to bind to circ-0002570 (**Figure 5B**). Then, overexpression of miR-587 distinctly suppressed the expressions of circ-0002570 in AGS cells, while miR-935 overexpression showed no change (**Figure 5C**). Thus, we chose miR-587 for subsequent experiments. The predicted binding sequence between miR-587 and circ-0002570 was shown in **Figure 5D**. To demonstrate the possible binding association between circ-0002570 and miR-587, a luciferase activity assay was conducted. We observed that co-transfection of miR-587 mimics and circ-0002570-WT distinctly decreased the luciferase activity (**Figure 5E**). Moreover, overexpression of circ-0002570 distinctly suppressed miR-587 expression, while circ-0002570 knockdown exhibited an opposite effect (**Figures 5F, G**). RIP assays also confirmed the combination between miR-587 and circ-0002570 (**Figure 5H**).

**Figure 5:** Circ-0002570 competitively sponged miR-587. **(A)** Representative FISH images indicated subcellular location of circ-0002570 in AGS cells. **(B)** Intersection of miRNAs predicted by circBank and CircInteractome databases. **(C)** RT-PCR examined the expression of circ-0002570 in AGS cells after miR-587 or miR-935 overexpression. **(D)** The binding sites of circ-0002570 and miR-587. **(E)** Luciferase reporter assay confirmed the molecular binding. **(F)** Overexpression of circ-0002570 resulted in the suppression of miR-587 expression. **(G)** Silence of circ-0002570 promoted the expression of miR-587. **(H)** RIP assays determined the combination between circ-0002570 and miR-587. *p < 0.05, **p < 0.01, ***p < 0.001.

### Circ-0002570 Regulates MiR-587 to Modulate VCAN in GC Cells

To explore the potential targeting genes of miR-587, we searched Starbase 2.0 and TargetScan database, and further performed comparation using the upregulated miRNAs in TGCA datasets. A total of eight overlapping targets were identified (**Figure 6A**). Then, we overexpressed miR-587 in AGS cells, finding that only VCAN expression was distinctly downregulated (**Figure 6B**). Thus, we chose VCAN for subsequent assays. Luciferase activity assays confirmed that VCAN was a target of miR-587 (**Figure 6B**). After miR-587 overexpression in AGS and SGC7901 cells, VCAN expression was distinctly decreased. However, when miR-587 expression was silenced, VCAN expression was distinctly increased (**Figure 6C**). Further Western blot assays also confirmed the above regulation (**Figure 6D**). These findings suggested VCAN as a target of miR-587. To further explore the association among circ-0002570, miR-587, and VCAN, we performed rescue experiments, finding that the distinct suppression of VCAN expression caused by circ-0002570-sh was reversed by the transfection of miR-587 inhibitor (**Figures 6E, F**). Then, we analyzed the expression and function of VCAN, finding that VCAN expression was distinctly increased in GC specimens compared with non-tumor specimens from our cohort and TCGA datasets (**Figures 7A–C**). Survival assays revealed that high circ-0002570 expression displays poor prognosis of GC patients based on the survival data of TCGA STAD cohort (**Figures 7D, E**). Then, we performed Data Mining Technology to delve into the possible functions of VCAN in tumor progression. Using GSVA, we found that the VCAN high-expression group was enriched in epithelial–mesenchymal transition (EMT)-related pathway, TGF-beta Signaling and Notch pathway, etc., which played a vital role in tumorigenesis (**Figure 7F**). KEGG and GO analysis indicated that VCAN was significantly related to several tumor-related pathways (**Figures 7G, H**). GSEA assays suggested a distinct correlation between VCAN and EMT and focal adhesion signaling, indicating their involvements in the metastatic activities of VCAN (**Figure 7I**). Finally, we further performed rescue experiments and observed that miR-587 knockdown or the transfection of pcDNA-VCAN reversed the distinct suppression of VCAN expression caused by circ-0002570-sh (**Figures 8A, B**). In addition, a series of functional assays revealed that miR-587 knockdown or the transfection of pcDNA-VCAN reversed the distinct suppression of the proliferation, invasion, and migration of AGS cells caused by circ-0002570-sh (**Figures 8C–F**). Overall, our findings suggested that circ-0002570 promoted GC progression by increasing VCAN expression *via* sponging miR-587.

**Figure 6:** VCAN is a target of miR-587. **(A)** Potential miRNA binding to circ-0002570. mRNA–miR-587 interaction was predicted by miRanda and targetscan. **(B)** RT-PCR for the levels of the potential candidates in AGS cells after miR-587 overexpression. Luciferase reporter assay confirmed the molecular binding. **(C, D)** The expression of VCAN at mRNA and protein in AGS and SGC7901 cells after miR-587 dysregulation. **(E, F)** RT-PCR and Western blot determined the expression of VCAN at mRNA and protein in AGS and SGC7901 cells transfected with NC-sh, circ-0002570-sh, or circ-0002570-sh+miR-587 inhibitor. *p < 0.05, **p < 0.01, ***p < 0.001.

**Figure 7:** The expression of VCAN in GC and its clinical significance. **(A, B)** VCAN expression was distinctly increased in GC specimens from our cohort and TCGA STAD cohort. **(C)** Western blot assays confirmed the increased levels of VCAN in GC specimens compared with non-tumor gastric specimens. **(D, E)** Survival assays based on VCAN expression using TCGA STAD cohort and kmplot online tool. **(F)** The bar plot showed the results of GSVA in the TCGA-STAD. **(G)** KEGG pathways significantly enriched. **(H)** The significantly enriched GO terms. **(I)** EMT and focal adhesion Signaling was enriched in the high-VCAN group. **p < 0.01, ***p < 0.001.

**Figure 8:** Circ-0002570 promoted GC progression *via* regulating miR-587/VCAN axis. **(A,B)** RT-PCR and Western blot determined the expression of VCAN in AGS cells transfected with NC-sh, circ-0002570-sh, circ-0002570-sh+miR-587 inhibitor, or circ-0002570-sh+pcDNA-VCAN. **(C)** CCK-8 assays, **(D)** Edu assays, **(E)** Colony formation assay, and **(F)** transwell assays of AGS cells after treatments. *p < 0.05, **p < 0.01, ***p < 0.001.

## Discussion

The identification of sensitive biomarkers is very important for the improvements of clinical outcome of GC patients (18). In recent years, growing studies highlighted the potential of circRNAs (CircRNA NALCN, Circ_0001588, and CircFAM73A) used as novel biomarkers for tumor patients, including GC (19–21). Here, the authors identified a novel GC-related circRNA, circ-0002570 whose back-splicing junctions was demonstrated by Sanger sequencing. We provided evidence that circ-0002570 was overexpressed in both GC specimens (GSE83521 and our cohort) and cells. Survival assays using TMA cohort demonstrated that patients with high circ-0002570 exhibited a poor prognosis of GC patients. Our findings suggested circ-0002570 as a possible prognostic biomarker for GC patients. However, the sample size was relatively small, and more samples were needed to further demonstrate the expressing pattern and clinical significance of circ-0002570 in GC.

It has been demonstrated that circRNAs could regulate the malignant phenotype of tumor by modulating tumor-related genes *via* various complex mechanisms (22). For instance, circ-BFAR was highly expressed in GC and its knockdown inhibits proliferation and glycolysis of tumor cells *via* increasing hexokinase 2 (23). Upregulated circ-100269 inhibits the growth and invasion of GC through inactivating the PI3K/Akt axis (24). Given that circ-0002570 was overexpressed in GC, we supposed it as an oncogenic circRNA. Then, we performed loss-of-function assays, finding that knockdown of circ-0002570 distinctly suppressed the proliferation, migration, and invasion of AGS and SGC7901 cells. *In vivo* assays also demonstrated the oncogenic effects of circ-0002570 on tumor growth. Our findings indicated that circ-0002570 facilitates GC progression, highlighting its potential use as a novel therapeutic target.

Transcripts with the same miRNA binding site, such as lncRNAs, mRNAs, and circRNAs, modulate the expressions of each other through competitively binding miRNAs (12, 25). The above ncRNAs and mRNAs form a multifaceted and accurate controlling network, namely, the ceRNA network (26). More and more studies have revealed that many circRNAs can act as miRNA sponges to modulate miRNA-targeting gene expressions in several types of cancers (27, 28). For instance, circSHKBP1 was shown to promote the metastasis of GC cells *via* sponging miR-582-3p to decrease HUR expression (29). Circular RNA circREPS2, a lowly expressed circRNA in GC, suppressed tumor growth by the regulation of RUNX3/β-catenin signaling *via* sponging miR-558 (17). In our study, FISH assays showed that circ-0002570 was mainly located in the cytoplasm of AGS cells, providing the probability of circ-0002570 acting as a ceRNA. Then, we confirmed that circ-0002570 could directly bind to miR-587. Previously, the dysregulation of miR-587 expression was reported in several tumors, and its overexpression was demonstrated to suppress the proliferation and metastasis of several tumor cells (30–32). We observed that overexpression of circ-0002570 suppressed the levels of miR-587, while its silence displayed an opposite effect. These findings together with previous results suggested that circ-0002570 may exhibit its oncogenic roles *via* sponging miR-587.

VCAN, an important extracellular matrix component, is a large aggregating chondroitin sulfate proteoglycan belonging to the lexicon family (33). It has been demonstrated that VCAN impacts cellular angiogenic, migrating, and adhering processes, thus positively influencing tissue maintenance and morphogenesis (34, 35). In recent years, growing studies suggested that VCAN was positively associated with tumorigenesis (36, 37). In GC, VCAN was reported to be highly expressed and promoted the proliferation and metastasis of GC cells (38, 39). In this study, we also found that VCAN was overexpressed in GC, and positively associated with tumor-related pathways. The prognostic value of VCAN was also confirmed using online data. These findings suggested VCAN as an oncogene in GC progression, which was consistent with previous studies (40). Then, we conducted bioinformatics, luciferase reporter, and Western blot, proving that VCAN was a downstream target gene of miR-587. Rescue experiments also confirmed that knockdown of circ-0002570 resulting in the distinct suppression of VCAN expression in AGS and SGC7901 was reversed by miR-587 inhibitor. More importantly, a series of functional assays demonstrated that circ-0002570 promoted GC progression by increasing VCAN expression through sponging miR-587.

## Conclusions

The present study provides some evidence that circ-0002570 is overexpressed in GC samples and that increased circ-0002570 predicted a poor prognosis for GC patients. Circ-0002570 exerts promoting effects on the proliferative, migrative, and invasive abilities of GC cells by increasing VCAN through sponging miR-587. Our data also suggest that circ-0002570 may act as a biomarker and a target for GC.

## Data Availability Statement

The datasets presented in this study can be found in online repositories. The names of the repository/repositories and accession number(s) can be found in the article/**Supplementary Material**.

## Ethics Statement

The studies involving human participants were reviewed and approved by The First Hospital of Lanzhou University. The patients/participants provided their written informed consent to participate in this study. The animal study was reviewed and approved by The First Hospital of Lanzhou University.

## Author Contributions

LY, M-MZ, and B-SW collected the patients’ data. LY, Y-NZ, and Q-LG drafted the manuscript. LY, M-MZ, and NZ revised the manuscript. NZ, B-SW, BL, and X-LZ analyzed and interpreted the data. X-LZ and CC made substantial contributions to the conception of the work. LY, Q-LG, and CC made substantial contributions to the design of the work and have revised the manuscript substantively. All authors contributed to the article and approved the submitted version.

## Funding

This work was supported by a grant from the Clinical Medical Science and Technology Development Foundation of Jiangsu University (JLY2021118) and Hospital Fund of the First Hospital of Lanzhou University (ldyyyn2019-32).

## Supplementary Material

The Supplementary Material for this article can be found online at: https://www.frontiersin.org/articles/10.3389/fonc.2021.733745/full#supplementary-material

## Conflict of Interest

The authors declare that the research was conducted in the absence of any commercial or financial relationships that could be construed as a potential conflict of interest.

## Publisher’s Note

All claims expressed in this article are solely those of the authors and do not necessarily represent those of their affiliated organizations, or those of the publisher, the editors and the reviewers. Any product that may be evaluated in this article, or claim that may be made by its manufacturer, is not guaranteed or endorsed by the publisher.
